# miR-211 alleviates ischaemia/reperfusion-induced kidney injury by targeting TGFβR2/TGF-β/SMAD3 pathway

**DOI:** 10.1080/21655979.2020.1765501

**Published:** 2020-05-13

**Authors:** Jinchun Shang, Shukai Sun, Lin Zhang, Fengyun Hao, Dianlong Zhang

**Affiliations:** a Department of Nephrology, The Affiliated Hospital of Qingdao University, Qingdao, Shandong, China; b Department of Clinical Lab, The Affiliated Hospital of Qingdao University, Qingdao, Shandong, China; c Department of Anesthesia, The Affiliated Hospital of Qingdao University, Qingdao, Shandong, China; d Department of Pathology, The Affiliated Hospital of Qingdao University, Qingdao, Shandong, China

**Keywords:** Hypoxia/reoxygenation, ischaemia/reperfusion, microrna, acute kidney injury, microrna-211, TGF-β

## Abstract

MicroRNA-211 (miR-211) is closely related to apoptosis and plays an important role in ischemia/reperfusion (I/R) injury. Whether miR-211 is involved in the protective effects in renal I/R injury is unknown. In this study, we evaluated the role of miR-211 in human tubular epithelial cells in response to hypoxia-reoxygenation (H/R) stimulation and I/R injury *in vitro* and *in vivo*. The results revealed that miR-211 was down-regulated and TGFβR2 was up-regulated in human kidney (HK-2) cells subjected to H/R. Luciferase reporter assay showed that TGFβR2 was a direct target of miR-211. Enforced miR-211 expression decreased H/R-induced HK-2 cell apoptosis and increased cell viability, and targeting miR-211 further increased H/R-induced HK-2 cell apoptosis and decreased cell viability. However, the effect of miR-211 was reversed by targeting TGFβR2 or enforced TGFβR2 expression in miR-211 overexpressing cells or miR-211 downexpressing cells. Moreover, we confirmed that miR-211 interacted with TGFβR2, and regulating TGF-β/SMAD3 signal. *In vivo* in mice, miR-211 overexpression ameliorates biochemical and histological kidney injury, reduces apoptosis in mice following I/R. On the contrary, miR-211 downexpressing promoted histological kidney injury and increased apoptosis in mice following I/R. Inhibition of miR-211 or miR-211 overexpression inhibited TGF-β/SMAD3 pathways or activated TGF-β/SMAD3 signal pathways *in vitro* and *in vivo*, which are critical for cell survival. Our findings suggested that miR-211 suppress apoptosis and relieve kidney injury following H/R or I/R via targeting TGFβR2/TGF-β/SMAD3 signals. Therefore, miR-211 may be as therapeutic potential for I/R- induced kidney injury.

## Introduction

Acute kidney injury (AKI) is a fatal syndrome and associated with high mortality. Ischemia/reperfusion (I/R) induced AKI results in renal tubular and endothelial cell injury, apoptosis and necrosis accompanied with leakage of tubular fluid and inflammation [1,2]. However, the mechanisms and effective treatment for renal I/R injury is limited [3].

MicroRNAs (miRNAs) are endogenous, small and noncoding RNAs that can induce its target mRNA degradation or bind to the 3′-untranslated region (3′-UTR) sequences of miRNAs to suppress mRNA translation [4]. By regulating miRNA-mediated gene expression, miRNAs can influence fundamental cellular processes such as the cell cycle, proliferation and apoptosis [5–8]. Recent studies have demonstrated that miRNAs play important roles in I/R-induced organ injury, such as myocardial injury [9,10], brain microvascular endothelial cells injury [11], small intestine injury [12] and hepatic Injury [13]. miRNAs also play important roles in I/R-induced kidney injury. For example, renal I/R injury stimulated miR-377 expression or inhibited miR-17-5p expression in the kidney. Targeting miR-377 or enforced miR-17-5p expression blocked I/R-induced oxidative stress and inflammation, and attenuated I/R-induced renal injury [14,15]. miR-21 inhibited inflammatory response and cell apoptosis in renal tubular epithelial cells exposure to I/R-induced AKI [16]. Given the role of majority of miRNAs in organ I/R injury, research on miRNAs helps to discover new targeted drugs or agents to regulate or prevent renal I/R injury [17–19].

miR-211 is reported to be as a pro-survival miRNA on the one hand [20], and also be as a pro-apoptotic miRNA on the other hand [21,22]. It has recently reported that enforced miR-204/miR-211 blocked Hmx1 expression and aggravated candidemia-induced kidney injury as reflected by improved renal glomerular filtration rate (GFR) [23]. Whereas miR-204/miR-211 knockout alleviated candidemia-induced kidney injury [23]. Takata et al. [24] reported that 14 miRNAs was upregulated, including miR-211 in hippocampal neuronal after transient whole-brain ischemia. Liu et al. [25] reported that OGD/R stimulation or MCAO reduced miR-211 expression in the PC12 cells in vitro or mice penumbra *in vivo*. Whereas, enforced miR-211 expression alleviated OGD/R-induced PC12 cell apoptosis, and vice versa *in vitro* [25]. However, the roles and mechanisms of miR-211 in renal I/R injury remained elusive.

Transforming growth factor-beta (TGF-β) is a pleiotropic multifunctional cytokine that regulates many cellular processes, such as cell growth, differentiation, apoptosis and cellular homeostasis [26]. Before exerting the biological effects within cells above, TGF-β first requires extracellular activation, namely binds to its type II receptor (TGFβR2) and promotes the phosphorylation [26]. Many miRNAs identified in various cancer types targeted TGF-β receptors, especially TGF-βR2, such as miR-21, miR-106b, miR-211 and miR-590 [27–31], all of which are frequently oncogenic [32]. TGF‐β/Smad3 signaling, which could be regulated by TGF-βR2, plays critical roles in a wide variety of biological processes including differentiation, inflammation, apoptosis, proliferation and epithelial‐mesenchymal transition (EMT) [33].

Here, we aimed to investigate the protective role and mechanism of miR-211 in renal epithelial NK-2 cells during H/R induced injury, and I/R induced kidney injury in mice. Our present findings demonstrated that enforced miR-211 inhibited apoptosis and protected NK-2 cell or kidney from H/R or I/R injury. We further demonstrated that miR-211 targeted TGFβR2, by which to activate the TGF-β1/Smad3 signaling pathway.

## Materials and methods

### Cell culture and hypoxia-reoxygenation (H/R) model

Human proximal tubular epithelial cells (HK-2) were purchased from American Type Culture Collection (ATCC, Manassas, VA, USA) and were maintain in Dulbecco’s modified Eagle’s medium (DMEM) supplemented with 10% fetal bovine serum (FBS) at 37°C and 5% CO_2_ in a humidified chamber.

To establish the H/R model, the 50–60% confluent HK-2 cells were subjected to a 24 h period of starvation, then the cells were placed in a sterile and sealed anaerobic bag containing 1% O_2_, 94% N_2_, 5% CO_2_ for 6 h. Then the hypoxic HK-2 cells were removed from the bag and transferred to 21% O_2_ and 5% CO_2_ conditions for 24 h. All the experimental methods have been approved by the research committee at the affiliated Hospital of Qingdao University.

### Generation of miR-211 overexpressing or downexpressing NK-2 cells

The miR-211 mimics, miR-211 inhibitors, their corresponding controls were synthesized by GenePharma (Shanghai, China). The sequences of **miR-211 mimic was**5′-UAACGACGAAUAACGCAAAAUGU-3′**; miR-211 inhibitors sequence was 5′-AGGCAAAGGATGACAAAGGGAA-3′**, and **the miControl sequence was 3ʹ-UCCGUUUCCUACAAAGCGGCAU-5ʹ.**

NK-2 cells were seeded at 2.5 × 10^5^ cells per well in 6-well plates and transfected with the miRNA mimics, or inhibitors to a final concentration of 100 nM by use of Lipofectamine 2000 (Life Technologies) according to the manufacturer’s instructions. After transfection for 6 hrs, the medium was replaced with fresh medium and cultured for another 48 h for further analysis. For the stable expression, fresh media containing 0.4 mg/ml G418 (Neomycin) was added at 2‐ to 3‐day intervals for 2–3 weeks. Stable lines were maintained in 0.2 mg/ml G418.

### Transient siRNA and plasmid transfection

Small interfering RNAs targeting TGFβR2 (TGFβR2 siRNA) and a corresponding negative control NC siRNA were purchased from RiboBio (Shanghai, China). The targeting sequence was **5′-AAGATGACCGCTCTGACATCA-3′, 5′-CTTATAGACCTCAGCGAC-3′)**. pCMV-TGFβR2 plasmid or empty vector DNA alone (pCMV) was purchased from OriGene Technologies, Rockville, MD. The siRNA and plasmid were transfected into the NK-2 cells by Lipofectamine™ 2000 reagent according to the manufacturer’s instructions. Briefly, the NK-2 cells or NK-2/miR-211 cells or NK-2/miR-211 inhibitor cells were seeded into 6‐well plate 24 h prior to transfection. Before transfection, cells were washed twice with serum-free Opti-MEM (Introgen Corp.). Then the Opti-MEM and Lipofectamine™ 2000 reagent were used to complex and transfect 100 nM TGFβR2 siRNA or pCMV-TGFβR2 or their control into cells according to the instructions of the manufacturer. After transfection for 48 h, the cells were collected for further analysis.

### Luciferase reporter assay

The targets of miR-211 and their potential binding regions were predicted using the TargetScan, miRanda and PicTar algorithms. The Wt TGFβR2-3′UTR and Mt TGFβR2-3′UTR constructs were purchased from Obio Technology (Shanghai, China). HEK293 cells were transfected with either WT or mutant TGFβR2-3′UTR constructs (100 ng) and miR-211 inhibitor or miR-NC inhibitor for 48 h using Lipofectamine 2000 (Invitrogen). Then the cells were harvested and assayed using the dual‐luciferase reporter assay system (Promega, Beijing, China) according to the manufacturer’s instructions. Each experiment was performed in triplicate.

### Quantitative RT-PCR

Total RNA was isolated from cell cultures using Trizol Reagent (Invitrogen, Shanghai, China) according to the manufacturer’s instruction. Complementary DNA (cDNA) was subsequently synthesized using the PrimeScript reverse transcription reagent Kit (Takara Biotechnology Co., Ltd.). U6 was selected as an endogenous control and reference gene of miR-211. The sequence for miR-211 was 5ˊ-CCGGAATTCCGGTTTTACAACACCCCATTTCACC-3ˊ,5ˊ-CGCGGATCCGCGCGAGCAACAGAGTAGAACAGG-3ʹ;**U6**: 5′-CTCGCTTCGGCAGCACA-3′. The RT-qPCR process was performed on an Applied Biosystems PCR7900 instrument using the protocol supplied by the manufacturer. The relative gene expression was calculated using the 2 − ΔΔCt method. All specimens were analyzed in triplicate.

### Western blot

Cells were lysed in lysis buffer containing 15 mM Tris/HCl pH 7.5, 120 mM NaCl, 25 mM KCl, 1 mM EDTA, 0.5% Triton 100 containing proteinase and phosphatase inhibitor cocktails (Sigma-Aldrich) at 4 °C for 40 min. Following centrifugation, the cell lysates were collected using 1 mL RIPA (Solarbio, Beijing, China) with 10 μL PMSF. Protein concentration was determined by BCA assay.

Protein lysates (50 µg) were resolved on 4–12% Novex Bis-Tris SDS-acrylamide gels (Invitrogen) and electrotransferred on Nitrocellulose membrane (Bio-Rad). The primary antibodies used in this study were anti- Smad3,anti-pSmad3, anti-TGFβR2 and anti-actin (Santa Cruz Biotechnology, Shanghai, China).

### Cell viability assayerence gene of

Cells were seeded in 96-well plates at a density of 5 × 10^3^ cells/well and left to recover for 24 h. Then the cells were transfected with TGFβR2 siRNA or pCMV-TGFβR2 or their controls using Lipofectamine 2000 as the manufacture’s instruction. After the cells were cultured at 37°C with 5% CO_2_ for 1–5 days, 10 μL of 3-(4,5-dimethylthiazol-2-yl)-2, 5-diphenyltetrazolium bromide solution(MTT) (5 mg/ml in PBS) was added to each well and the plates were incubated for another 4 h. The formazan products of MTT were dissolved and the absorbance was measured at 490 nm using microplate reader (Varioscan Flash; Thermo Fisher Scientific). Experiments were performed in duplicate.

### Terminal deoxynucleotidyl transferase-mediated dUTP nick end-labeling (TUNEL) staining in vitro

TUNEL staining was used to detect apoptosis-specific nuclear DNA fragmentation. Briefly, cells on coverslip were fixed in 4% paraformaldehyde for 60 min at room temperature. Then the cells were incubated with 50 μl proteinase K and 50 μl Strep-DAB/Fluor solution, respectively. After that, the fixed cells were then stained using the TACS2 TdT-DAB/Fluor in situ apoptosis detection kit (Trevigen, Gaithersburg, Shanghai, China). Finally, cells were analyzed under a fluorescence microscope (Nikon Corporation, Tokyo, Japan). The number of positive cells was counted in five microscopic fields from each slide.

### Rat model for renal injury and treatment of rats with miR-211 mimics or miR-211 inhibitors

**The femal mice (12–16 g) were obtained from Shanghai Experimental Animal Center (Shanghai, China). All animal feeding and operations were in accordance with experimental animal ethics and animal welfare. The left renal pedicle was clamped for 45 min** at 24 ± 0.5°C**, and the right kidney was either left intact for control purposes. After the operation, the rats were placed in the normal environment, and their vital signs observed. Animals were sacrificed at 72 h of reperfusion and kidneys were harvested.**

***In vivo*, miR-211 mimics or miR-211 inhibitors were administered (100 mg/kg) with Entranster™ (Engreen Biosystem Co. Ltd., Beijing, China) and intravenously injected through the tail vein 24 h before ischemia in sham and ischemia groups. After kidney I/R for 3 days, the relative index of renal function and miR-211 and relative protein expression were determined.**

**For TUNEL assay, renal tissue was fixed in 4% phosphate-buffered formalin, and 3 μm sections of paraffin-embedded kidneys were used. TUNEL assay was performed using the TACS2 TdT-DAB/Fluor in situ apoptosis detection kit (Trevigen, Gaithersburg, Shanghai, China). Positive cells were counted (× 200).**

### Assessment of serum creatinine (Cr)

Blood samples were drawn via cardiac puncture. Plasma creatinine was measured with a biochemical autoanalyzer (TBA-200FR; Shanghai, China).

### Histology

**Tissues were fixed, dehydrated, paraffin embedding and the 4 µm sections were prepared and stained with H.E using the standard methods. The tissue injury scores were quantified in a blinded fashion as follows: tubular dilatation, vacuolization, tubular cell necrosis, loss of brush border, interstitial edema and inflammatory cell infiltration.**

### Statistical analyses

Data are expressed as mean ± standard error of the mean (SEM). Statistical analysis was performed using the Student’s t-test or one way analysis of variance (ANOVA) with Dunnett’s multiple comparison test. Analysis for significance was performed with GraphPad Prism 6.0 (GraphPad Software Inc.). P values < 0.05 were considered significant.

## Results

### miR‐211 expression in HK-2 cells after H/R stimulation

HK-2 cells were subjected to H (6 h)/R (24 h), the endogenous miR‐211 expression was detected by qRT‐PCR. A shown in Figure 1(a), 85% decrease of miR‐211 expression was observed in the H (6 h)/R (24 h) treated HK-2 cells, and no significant change was observed in the normoxic condition groups.

**Figure 1.** Overexpression of miR-211 aggravated H/R-induced apoptosis in NK-2 cells

(a) Expression of miR-211 was detected in NK-2 cells or NK-2/miR-211 mimics cells following H/R by qRT-PCR assay. (b) CCK-8 method was employed to detect cell viability after the treatment for 24 h-120 h. (c) Representative images of TUNEL staining to measure apoptosis of HK-2 cells. Data shown are means ± SE for n = 3 independent experiments. Student’s t test,*P <.05;**P < 0.01.

### Enforced miR-211expression alleviates cell apoptosis induced by H/R stimulation

HK-2 cells were treated with miR‐211 mimic or negative control (miR-NC), then the cells were subjected to H (6 h)/R (24 h). As shown in Figure 1(a), cells transfected with the miR‐211 mimic showed more than 7.4 fold increase of miR-211 expression. No significant change was found in the NC transfected HK-2 cells.

Compared with the normoxic condition group, H/R treatment decreased cell viability (Figure 1(b)) and increased HK-2 cell apoptosis (Figure 1(c)). However, enforced miR-211 expression increased H/R-induced cell viability (Figure 1(b)) and decreased H/R-induced cell apoptosis (Figure 1(c)). The miR-NC transfection has no significant effect on H/R-induced cell apoptosis and cell viability (Figure 1(b,c)).

### *Targeting miR-211 aggravated H/R-induced cell apoptosis* in vitro

To consolidate the role of targeting miR-211 on H/R-induced cell viability and apoptosis, NK-2 cells were transfected with miR-211 inhibitor or control NC inhibitor. As shown in Figure 2(a), miR-211 inhibitor further suppressed intracellular miR-211 expression in the NK-2 cells following H/R treatment compared to the NC inhibitor. Targeting miR-211 significantly aggravated H/R-induced cell injury, as evidenced by decreased cell viability (Figure 2(b)) and increased cell apoptosis (Figure 2(c)).

**Figure 2.** Targeting miR-211 increased H/R-induced cell apoptosis in NK-2 cells. (a) Expression of miR-211 was detected in NK-2 or NK-2/miR-211 inhibitor cells following H/R by qRT-PCR assay. (b) CCK-8 method was employed to detect cell viability after the treatment for 24 h-120 h. (c) Representative images of TUNEL staining to measure apoptosis of HK-2 cells. Data shown are means ± SE for n = 3 independent experiments. Student’s t test,*P <.05

### TGFβR2 is the direct target of miR-211

The targets of miRs and their potential binding regions were predicted using the TargetScan, miRanda and PicTar algorithms. All three algorithms predicted miR-211 as a regulator of TGFβR2. As Figure 3(a) shows, there was one hypothetic miR-211 binding site in the TGFβR2 3′‐UTR. To determine whether the TGFβR2 3′‐UTR was the functional target of miR-211, we examined the reporter activity of the wild-type (Wt) 3′-UTR sequences of TGFβR2. As shown in Figure 3(b), miR‐211 inhibitor resulted in decreased miR-211 expression in the NK-2 cells. MiR‐211 inhibitor increased the luciferase activity in the TGFβR23′‐UTR‐WT transfected NK-2 cells, but not in those with TGFβR23′‐UTR‐MT transfected NK-2 cells (Figure 3(c,d)). These results support the targeting relationship between miR-211 and TGFβR2 at the gene level. We also confirmed that miR-211 downregulated TGFβR2 protein expression in NK-2 cells (Figure 3(e)), which was consistent with the result of the luciferase reporter assay (Figure 3(c)).

**Figure 3.** Interaction between miR‐211 and TGFβR2 in NK-2 cells. (a) The predicted site in TGFβR2 3′‐UTR for binding miR‐211. (b) Expression of miR-211 was detected in NK-2/miR‐211 inhibitor cells or NK-2/miR‐NC cells by qRT-PCR assay. (c) Luciferase reporter assay of NK-2 cells transfected with the TGFβR2 3′‐UTR‐WT or TGFβR2 3′‐UTR‐M in the binding sites. Differences were observed when miR‐211 inhibitor was added, and miR‐NC was used as the control. (d) TGFβR2 protein was detected by western blot assay in NK-2 cells transfected with miR‐211 inhibitor or miR‐NC. (e) miR‐211 inhibitor could reverse the TGFβR2 protein expression by TGFβR2 siRNA transfection by Western blot analysis. Data shown are means ± SE for n = 3 independent experiments. Student’s t test,*P < 0.01

### miR-211 Inhibits TGF-β/SMAD signaling in H/R induced NK-2 cells

TGFβR2 is a canonical reporter, which regulates TGF‐β/Smad3 signaling and phosphorylates Smad3. We next investigated whether miR-211 regulates TGFβR2 and TGF-β/SMAD signal to influence cell apoptosis and cell viability. Following H/R in the NK-2 cells, the expression of TGFβR2 protein was increased and the expression of phosphorylated Smad3 (p-SMAD3) was dramatically decreased by western blot analysis (Figure 4(a)). However, enforced miR-211 expression by miR-211 mimics transfection decreased TGFβR2 expression and increased p-SMAD3 levels (Figure 4(a)). While co-transfected with pCMV6-TGFβR2 and miR-211 mimics restored p-SMAD3 protein expression in H/R -induced NK-2 cells (Figure 4(b)). Furthermore, TGFβR2 overexpression decreased cell apoptosis in H/R-induced NK-2/miR-211 mimics cells. Targeting TGFβR2 by TGFβR2 siRNA blocked H/R-induced TGFβR2 expression and increased p-SMAD3/SMAD3 levels (Figure 4(c)). In addition, targeting TGFβR2 inhibited H/R-induced NK-2 cell apoptosis (Figure 4(d)).

**Figure 4.** MiR-211 overexpression inhibited H/R induced NK-2 cell apoptosis through alleviating TGFβR2/TGF-β/SMAD signaling. (a) H/R induced NK-2 cells were transfected with miR-211 mimic or control NC and the protein levels were analyzed by Western blot assay. (b) H/R induced NK-2 cells were co-transfected with miR-211 mimic and pCMV6-TGFβR2 (TGFβR2) or pCMV6 and the protein levels were analyzed by Western blot assay. (c) H/R induced NK-2 cells were transfected with TGFβR2 siRNA or control siRNA and the protein levels were analyzed by Western blot assay. (d) Cell apoptosis was detected in H/R induced NK-2 cells transfected or co-transfected with TGFβR2 siRNA, pCMV6-TGFβR2, miR-211 mimic and their controls. Data shown are means ± SE for n = 3 independent experiments. Student’s t test, *P < 0.01

### Targeting miR-211 promotes TGF-β/SMAD signaling H/R induced NK-2 cells in vitro

NK-2 cells was transfected with miR-211 inhibitor or NC inhibitor in the NK-2 cells, then exposure to H/R stimulation. After NK-2 cells were transfected with miR-211 inhibitor, TGFβR2 expression was further increased and p-SMAD3/SMAD3 levels was completely blocked in H/R induced NK-2 cells by WB analysis (Figure 5(a)). Targeting TGFβR2 with TGFβR2 siRNA blocked miR-211 inhibitor induced TGFβR2 expression (Figure 5(a)) and reduced cell apoptosis (Figure 5(a)) in H/R induced NK-2 cells. In addition, co-transfected with TGFβR2 siRNA and miR-211 inhibitor restored H/R induced p-SMAD3 protein expression (Figure 5(b)). These findings suggest that targeting miR-211 resulted in TGFβR2 upregulation to modulate TGF-β/SMAD signaling in H/R induced NK-2 cells.

**Figure 5.** Targeting miR-211 promoted H/R induced NK-2 cell apoptosis through activating TGFβR2/TGF-β/SMAD signaling. (a) H/R-induced NK-2 cells were transfected with miR-211 inhibitor or NC inhibitor or TGFβR2 siRNA and the protein levels were analyzed by Western blot assay. (b) Cell apoptosis was detected in H/R induced NK-2 cells transfected or co-transfected with TGFβR2 siRNA, miR-211 inhibitor and their controls. Data shown are means ± SE for n = 3 independent experiments. Student’s t test,*P < 0.05;**P < 0.01

### *The protective role of miR-211 on I/R injury* in vivo

**To investigate the roles of miR-211 in response to I/R, we analyzed miR-211 expression under ischemia/reperfusion (I/R) conditions *in vivo*. We found that I/R decreased miR-211 expression** (Figure 6(a)). **The kidney injury was assessed by histology and Cr level. As the results indicated, miR-211 inhibitor further reduces the miR-211 level caused by I/R** (Figure 6(a)). **Furthermore, renal function is exacerbated in animals subject to miR-211 inhibitor compared with scramble control** (Figure 6(b)). **Kidney injury was also exacerbated analyzed based on PAS staining** (Figure 6(c)). **However, miR-211 mimics reversed I/R induced miR-211 downregulation** (Figure 6(a)) **and reduced renal function in animals subject to I/R** (Figure 6(b,c)). **The control miR-NC or anti-miR-NC has no significant effect on miR-211 expression and renal function (data not shown)**.

**Figure 6.** miR-211 protects mice kidney from I/R-induced renal injury. miR-211 mimics or miR-211 inhibitors (100 mg/kg) was intravenously injected through the tail vein 24 h before ischemia in sham and ischemia groups. After kidney I/R for 3 days, the miR-211 expresssion was detected by qRT-PCR assay in kidney tissues (a), Cr was detected in the blood of the mice (b), pathological score was shown (c), TGFβR2 and p-Smad3 protein was detected by western blot, cell apoptosis was detected by TUNEL staining (d). *P < 0.05;**P < 0.01; ***P < 0.001

**In addition, we investigated the effect of miR-211 on TGF-β/SMAD3 signal after I/R. I/R induced TGF-β/SMAD3 expression in the kidney, and knockdown of miR-211 increased the expression of TGF-β/SMAD3 in IR-challenged kidney** (Figure 6(d)). **And miR-211 overexpression decresed the TGF-β/SMAD3 expression in I/R-challenged kidney** (Figure 6(d)). **TUNEL staining showed that miR-211 mimics inhibited I/R-induced cell apoptosis, and miR-211 inhibitor increased I/R-induced cell apoptosis in the kidney** (Figure 6(e)).

## Discussion

Hypoxia plays an important role in I/R injury including renal I/R injury. Cumulative studies have confirmed that miRNAs play an important regulatory role in hypoxic responses [34–36]. Emerging evidence suggests that miRNAs contribute to regulating processes involved in I/R injury [37–39]. Prevention and treatment of I/R injury are an important area of research in myocardial infarction, stroke, and acute kidney injury [40].

miR-211 has reported to reduce neuron apoptosis in a neonatal rat model of hypoxic-ischemic injury [41], and alleviates focal cerebral ischemia-reperfusion injury in rats [25,42]. In this study, we found that miR-211 was downexpressed both in proximal renal tubular cells subjected to H/R and in mice kidney subjected to I/R injury. Furthermore, enforced miR-211 expression protected NK-2 cells from H/R injury *in vitro*. This study also provides further evidence for a functional role of miR-211 in the recovery from renal I/R injury *in vivo*. Mechanistically, H/R or I/R induced cell or renal injury by downregulation of miR-211, resulting in increased cell apoptosis and kidney injury. Enforced miR-211 expresssion can reversed H/R or I/R induced cell or renal injury. And downregulation of miR-211 further aggravated H/R or I/R-induced cell apoptosis and renal injury. Therefore modulation of miR-211 might be a valuable therapeutic option in the treatment of patients with renal I/R injury.

The molecular mechanism involving miR-211 is still unknown. Emerging evidence suggests that upon stimulation, TGF**β**R2 first binds to TGF-β, resulting in auto-phosphorylates and triggering a cascade response that ultimately results in gene regulation of a series of genes involved in different pathophysiological processes [43]. In this study, TGFβR2 was identiﬁed as a functional target of miR-211. Enforced miR-211 expression inhibited H/R-induced NK-2 cell apoptosis through degradation of TGFβR2 transcription and activating TGF-β/SMAD3 signaling. On the contrary, downexpressing miR-211 further promoted H/R-induced NK-2 cell apoptosis through promotion of TGFβR2 transcription and inactivating TGF-β/SMAD signaling.

TGFβR2 is a transmembrane receptor of the TGF-β/SMAD signaling which induces SMAD2/3 phosphorylation and inhibits cell apoptosis [44]. In this study, the expression of p-SMAD3 was signiﬁcantly reduced in H/R treated NK-2 cells. Furthermore, miR-211 inhibitor or TGFβR2 overexpression further reduced p-SMAD3 expression in the H/R stimulated NK-2 cells. However, Knockdown of TGFβR2 or miR-211 mimics resulted in a increase of p-SMAD2/3 levels in the H/R treated NK-2 cells. This suggested that H/R regulates miR-211/*TGFBR2*/TGF-β/SMAD3 signaling pathway to induce cell apoptosis *in vitro*.

Our data *in vivo* support the above results *in vitro*. miR-211 was downregulated in an experimental model of I/R kidney in mice. Targeting miR-211 *in vivo* further increased cell apoptosis and promotes renal I/R injury as well as kidney function in mice. However, miR-211 *in vivo* resulted in protection against endothelial and tubular epithelial apoptosis and inhibited renal I/R injury and protected kidney function in mice. Moreover, we identify the underlying molecular mechanisms by analyzing miR-211,TGFβR2 and TGF-β/SMAD3 signal and found that miR-211 protected kidney from I/R injury through TGFβR2/TGF-β/SMAD3 signal.

## Conclusion

In conclusion, H/R and I/R condition down-regulated miR-211 expression and induced miR-211-dependent cell apoptosis in NK-2 cells *in vitro* and mice kidney *in vivo*. The enforced miR-211 expression inhibited H/R induced NK-2 cell apoptosis and I/R-induced renal injury by regulating TGFβR2/TGF-β/SMAD signaling pathway. Therefore, miR-211 can be potentially therapeutic target for the treatment renal I/R injury.

## Highlights

1. Hypoxia/reoxygenation (H/R) downregulated miR-211 expression in the HK-2 cells *in vitro*

2. Renal ischemia/reperfusion (I/R) downregulated miR-211 expression in the mice kidney *in vivo*

3. Enforced miR-211 decreases H/R-induced cell apoptosis via regulating TGFβR2/TGF-β/SMAD3 signal

4. Enforced miR-211 protects I/R-induced renal injury via regulating TGFβR2/TGF-β/SMAD3 signal
